The article "Intervertebral Disc Degeneration and Low Back Pain Depends on Duration and Magnitude of Axial Compression" was published in 2022. Journal: Oxid Med Cell Longev.

# Intervertebral Disc Degeneration and Low Back Pain Depends on Duration and Magnitude of Axial Compression

**DOI:** 10.1155/2022/1045999

**Published:** 2022-04-29

**Authors:** Jitian Li, Yan Ma, Yucheng Jiao, Libo Xu, Yage Luo, Jiancheng Zheng, Xingkai Zhang, Zhe Chen

**Affiliations:** ^1^Henan Luoyang Orthopedic Hospital (Henan Provincial Orthopedic Hospital), Henan Provincial Orthopedic Institute, Zhengzhou 450000, China; ^2^Henan University of Chinese Medicine, Zhengzhou 450046, China; ^3^Department of Orthopeadics, Ruijin Hospital, Shanghai Jiaotong University School of Medicine, Shanghai 200025, China; ^4^Shanghai Key Laboratory for Prevention and Treatment of Bone and Joint Diseases with Integrated Chinese-Western Medicine, Shanghai Institute of Traumatology and Orthopedics, Ruijin Hospital, Shanghai Jiaotong University School of Medicine, Shanghai 200025, China

## Abstract

**Purpose:**

The pathological role of axial stress in intervertebral disc degeneration (IDD) is controversial, and there was no quantified study until now. Here, we tried to clarify the correlation between IDD or low back pain (LBP) and axial stress at different duration and magnitude in vitro and in vivo.

**Method:**

In vitro, the gene expression of aggrecan, matrix metalloproteinase-3 (MMP3), calcitonin gene-related peptide (CGRP), and substance P (SP) was measured when nucleus pulposus cells (NPCs) were compressed under gradual severity. In vivo, a measurable Ilizarov-type compression apparatus was established for single coccygeal (Co) intervertebral disc (IVD) compression of Co7-8 in mouse. Gradient stress was placed at 0.4 Mpa (mild), 0.8 Mpa (moderate), and 1.2 Mpa (severe) for three days to investigate the effect of the magnitude of axial stress. Additionally, mild compression with 3, 7, and 14 days was used to determine the effect of the duration of axial stress. Subsequently, we evaluated the severity of IDD and LBP by radiological X-ray film; histological examination with H&E staining; immunohistochemical analysis with collagen II, aggrecan, and CGRP staining; and western blot analysis with collagen II, aggrecan, MMP-3, and interleukin-1*β* (IL-1*β*).

**Results:**

When NPCs suffered gradual increased mechanical stress, the cells exhibited gradual downregulated expression of extracellular matrix (ECM)-related gene of aggrecan, upregulated expression of IDD-related gene of MMP3, and LBP-related gene of CGRP and SP. In the meantime, with different magnitudes of axial stress, the IVD showed progressively severe IDD and LBP, with gradual narrowing intervertebral height, destruction of IVD anatomy, decreased ECM, and increased catabolic factors and proalgesic peptides.

The article "Intervertebral Disc Degeneration and Low Back Pain Depends on Duration and Magnitude of Axial Compression" was published in 2022. Journal: Oxid Med Cell Longev.

**Conclusion:**

Axial compression is one of the critical pathological factors to cause IDD and LBP, and there was a strong positive correlation depended on the duration and magnitude of compression.

## 1. Introduction

Intervertebral disc degeneration (IDD) is a serious health problem worldwide. Generally, IDD is an initiation for serious spine diseases, such as intervertebral disc (IVD) herniation, sciatica, and spondylolisthesis, among others. Although there are plenty of methods to treat these diseases, there is a lack of strategies to prevent IDD. A common challenge that surgeons and researchers face is how to effectively prevent IDD.

There are several etiologies that are thought to initiate and deteriorate IDD [1], such as axial or shear stress [2], gene diversity [3], biochemical environment change [1], or low-virulence anaerobic bacterial infection [4]. Although axial stress was considered as the main factor for IDD, some research does not support the pathological role of axial stress. For example, a classical cohort study with monozygotic twin pairs suggested that physical activities explained only 2% to 7% of IDD, according to multivariate analyses [5]. Also, an epidemiological study found that the association between physical activity and lumbar spondylosis was weak [6].

In the meantime, IDD also had a strong correlation with low back pain (LBP). Plenty of previous epidemiological studies suggested that IDD was a direct factor to cause LBP, which was also named as discogenic LBP [7]. LBP would significantly reduce quality of life and increase psychological burden in patients and approximately one-quarter of US adults reported having LBP lasting at least 1 whole day in the past 3 months, and 7.6% reported at least 1 episode of severe acute low back pain within a 1-year period [8]. Thus, effective methods to prevent and treat IDD and discogenic LBP are urgent for researchers all over the world.

To elucidate the pathological role of mechanical stress in IDD and LBP, the nucleus pulposus cells (NPCs) were compressed in vitro, and related genes were quantified. In addition, we establish a creditable animal model to verify the axial stress as the etiology for IDD, especially quantifiable models to investigate the potential dose-response manner at different duration and magnitude levels. Moreover, the novel compression IVD model we proposed provided a measurable and comparative apparatus for IDD studies in mice, which was useful in gene-knockout animals. The results would provide adequate evidence to confirm that axial stress is the key etiology for IDD.

## 2. Methods and Materials

### 2.1. Animals and Surgery

Male, 8-week-old C57BL/6 mice were used in this study. All of the animal experiments performed were approved by the Institute of the Animal Care and Use Committee of Ruijin Hospital, Shanghai Jiao Tong University School of Medicine and followed the National Institutes of Health guidelines for the care and use of laboratory animals (NIH Publications No. 8023, revised 1978).

The article "Intervertebral Disc Degeneration and Low Back Pain Depends on Duration and Magnitude of Axial Compression" was published in 2022. Journal: Oxid Med Cell Longev.

The animal model followed our previous report [9]. In brief, sodium pentobarbital (2.5%) was used, via intraperitoneal injection, for anesthetization in order to perform coccygeal (Co) IVDs of C7-8 that were identified with X-ray examination as the target IVDs. As depicted in Figure 1, an Ilizarov-type compression apparatus (Shanghai Yeyu Biotech Inc., Shanghai, China) was placed to induce axial compression for Co7-8. In brief, two cross 0.4-mm diameter wires were inserted percutaneously into each of the 7th and 8th coccygeal vertebrae. The two wires were perpendicular to each other and parallel to the endplates of vertebrae. Then, the two wires were attached to the specific manufactured two resin rings that were connected longitudinally with four threaded rods. Finally, axial loads were applied using calibrated springs installed over each rod, which were tightened from the distal side. A thin-film pressure sensor was placed between the springs and rings to detect the pressure produced by springs, and the force between each spring and the ring was measured by sensors in turn and fixed at the same level. The pressure is measured daily and guaranteed at the initial strength via fixing the springs. After surgery, all mice were placed on a heating pad for recovery, and saline was administered subcutaneously to prevent dehydration. Oral NASIDs drug was used if the mice had any symptoms of pain.

In this study, axial compression pressure was fixed at 0.4, 0.8, and 1.2 Mpa at different compression severities. Previous studies have estimated that the stress for mouse to lift the tail, against gravity, was in the range of 0.4 MPa, which is comparable to that in humans during an upright stance, and thus, we calibrated this as mild compression [10]. We then fixed twice of the 0.4 Mpa (i.e., moderate compression) and three times of 1.2 Mpa (i.e., severe compression), each of which corresponded to spinal force in human activities of walking and lifting a moderate weight [10]. In sham surgery animals, only the rings and rods were installed, and no springs were placed in the rods.

To analyze the magnitude of axial compression for IDD, five groups of normal, sham surgery, mild compression, moderate compression, and severe compression at 3 days were established. Then, 5 groups of normal, sham surgery animals at 3, 7, and 14 days with mild compression were established to analyze the duration of axial compression for IDD.

The article "Intervertebral Disc Degeneration and Low Back Pain Depends on Duration and Magnitude of Axial Compression" was published in 2022. Journal: Oxid Med Cell Longev.

### 2.2. Human Nucleus Pulposus Cells (NPCs) Extraction and Treatment

After being harvested from surgery, samples were digested and cultured as previously reported [9, 11]. Before compression, NPCs at the 2^nd^ passage were harvested and mixed with Corning matrix gel (Cat No. 356234, Corning, USA) for three days. For compression treatment, we set compression of 20 kPa for a duration of 0, 2, 4, 6, and 12 hours with a Flexcell FX-5000 Tension System.

### 2.3. Real-Time Quantitative PCR

RNA extraction and synthesis of cDNA was conducted using a specific kit of Takara Premix Taq (Cat no. R004A, Takara Bio Inc., Shiga, Japan.) according to the manufacturer's instructions. An ABI 7500 Sequencing Detection System (Applied Biosystems, CA, U.S.) was employed for qRT-PCR detection and analysis using the SYBR Premix Ex Tag Kit (Cat no. RR420A, Takara, Shiga, Japan). The cycling conditions were set as follows: 40 cycles of denaturation at 95°C for 5 s and amplification at 60°C for 24 s. *GAPDH* served as a housekeeping gene, and all reactions were run in triplicate. The primer sequences (Sangon Biotech, Shanghai, China) used in this study were as follows:

human *GAPDH* forward 5′- CTTAGCACCCCTGGCCAAG-3′;

reverse 5′- TGGTCATGAGTCCTTCCACG-3′;

human *SUBSTANCE P*: forward 5′- GCAGAAGAAATAGGAGCCAATG-3′;

reverse 5′- CATAAAGAGCCTTTAACAGGGC-3′;

human *AGGRECAN*: forward 5′- GATCCTTACCGTAAAGCCCATC-3′;

reverse 5′ CTCCAGTCTCATTCTCAACCTC-3′;

human *MATRIX METALLOPROTEINASE-3* (*MMP-3)*:

forward 5′- GGCAAGACAGCAAGGCATAGAGAC-3′;

reverse 5′ ACGCACAGCAACAGTAGGATTGG-3′.

Human *CALCITONIN GENE RELATED PEPTIDE*(*CGRP*):

forward 5′- CAGGACTATGTGCAGATGAAGG -3′;

reverse 5′ CTCTCTTCTGGGCAATGATTCT-3′.

Target gene expression was normalized to the expression of *GAPDH* using the 2^-△△Ct^ method. All data were then normalized to the average of the control group.

### 2.4. Histology

For histological observation, the IVDs were initially fixed with 4% formaldehyde for 24 hours. Routine paraffin embedding was performed for all of the samples, and they were sectioned to 5 *μ*m. Routine hematoxylin-eosin (H&E) staining was conducted following the manufacturer's instructions. The stained samples were observed and photographed under a microscope (Axio, Carl Zeiss, Oberkochen, Germany). To evaluate degree of IDD, we followed the protocol of modified Thompson grade scale [12], and two authors who were blinded to the group conducted the evaluation separately.

### 2.5. Immunohistochemistry (IHC)

IVDs were fixed with 4% paraformaldehyde for 24 h and then decalcified using 10% ethylenediaminetetraacetic acid (EDTA) for 1 month. After routine embedding, sectioning, and deparaffinizing, the sections were incubated with antimouse collagen II antibody (cat. no. GB11021, Servicebio Inc., Shanghai, China) and antimouse aggrecan antibody (cat. no. GB11373, Servicebio Inc., Shanghai, China) at 4°C overnight. A specific IHC kit (cat. no. K5007, Agilent DAKO Inc., CA, US) was used for the whole process following manufacturer's protocol. Nuclei were counterstained with hemalum (cat.no.G1004, Servicebio Inc., China). The stained samples were observed and photographed under a microscope (Axio, Carl Zeiss, Oberkochen, Germany).

The article "Intervertebral Disc Degeneration and Low Back Pain Depends on Duration and Magnitude of Axial Compression" was published in 2022. Journal: Oxid Med Cell Longev.

### 2.6. Western Blotting Analysis

In the western blot analysis, the samples were incubated with antimouse collagen II (cat. no. ab34712, Abcam, Cambridge, UK), antimouse aggrecan (cat. no. ab3778, Abcam, Cambridge, UK), antimouse MMP3 (cat. no. AF7482, Beyotime Biotech Inc., Shanghai, China), and antimouse IL-1*β* (cat. no. ab200478, Abcam, Cambridge, UK) overnight. They were then incubated with horseradish peroxidase-conjugated secondary antibody and goat antirabbit IgG (cat. no. CW0103s; CW Bio, Beijing, China) at room temperature for 2 h. *β*-Actin were used as the internal controls. The bands were visualized using chemiluminescence (Pierce Biotechnology Inc., IL, USA) and analyzed using a Fusion FX7 (Vilber Lourmat, Marne-la-Vallée, France).

### 2.7. Radiological Evaluation

For radiological evaluation at the end of following-up, animals were anaesthetized using a 2.5% sodium pentobarbital to keep them in a fixed position and then placed in a prone position. Data were acquired using a low-energy X-ray machine (Faxitron MX-20, IL, USA) at an exposure time of 30 s (30 kV).

### 2.8. Statistics

All of the data are presented as mean ± SD. For multiple group analysis, One-way ANOVA, with post hoc of Tukey's HSD test, was used. For all of the statistical tests, we considered *p* < 0.05 to be statistically significant.

## 3. Results

### 3.1. Gradient Mechanical Compression of NPCs Induced Gradual IDD and LBP In Vitro

As depicted in Figure 1, the NPCs suffered the gradient mechanical stress at 0 h, 2 h, 4 h, 6 h, and 12 h, and then the cells exhibited gradual downregulated expression of ECM-related gene of aggrecan, upregulated expression of IDD-related gene of MMP3, and LBP-related gene of CGRP and SP, with a time-response manner. Thus, we made conclusion that gradient mechanical stress was a critical factor to cause IDD and LBP, at least in vitro study.

### 3.2. Gradient Mechanical Compression Magnitude Induced Gradual Severer IDD In Vivo

To investigate our hypothesis, we developed an Ilizarov-type compression apparatus for single level of coccygeal IVDs. As depicted in Figure 2, the compression pressure was measurable and comparable, and gradient compression duration and magnitude could be fixed.

The article "Intervertebral Disc Degeneration and Low Back Pain Depends on Duration and Magnitude of Axial Compression" was published in 2022. Journal: Oxid Med Cell Longev.

Three days after compression, the severity of IDD was assessed with radiological and histological confirmations. As depicted in Figure 3(a) of X-ray examination, the intervertebral height of targeted IVDs gradually narrowed. With the result of histological examination in Figure 3(b), the IVDs showed normal appearance, indicating aggrecan-rich, bulging nucleus pulposus with rare proliferated chondrocytes and no clefts, and organized annulus fibrosus as discrete fibrous lamellae in sham surgery animals. Mild compression caused slight degeneration of IVD, as shown by growth of small, amorphous fibrosus tissue and slight proliferated chondrocytes in nucleus pulposus, and slight disorganized annulus fibrosus. IVD with moderate compression showed as bulged nucleus pulposus replaced by large fibrosus tissue and proliferated chondrocytes and focal lamellar disruptions of disorganized annulus fibrosus. Severe compression induced serious degeneration of IVD, as shown by consolidated fibrous tissue in nucleus pulposus with disappearance of notochordal cells and the numerous levels of proliferated chondrocytes, lamellar disruptions of disorganized annulus fibrous, and radial clefts through nucleus pulposus and annulus fibrosus. Based on the modified Thompson grade scale, the IDD grade for the sham surgery, mild, moderate, and severe compression groups were 1, 2, 4, and 5, respectively, suggesting gradually severer IDD under a gradient compression pressure.

Based on radiological and histological analysis, we further explored the effect of gradient compression magnitude for content of extracellular matrix (ECM). As depicted in Figure 3(c), western blot analysis suggested the loss of ECM in a dose-response manner, showing a significant decrease of aggrecan and collagen II, in addition to an increase of catabolic factors of interleukin-1*β* (IL-1*β*) and matrix metalloproteinase-3 (MMP-3). In the meantime, IHC analysis also verified the gradually loss of ECM in Figure 3(d) . Altogether, these results suggest that gradient compression magnitude resulted in gradual IDD.

### 3.3. Increased Mechanical Compression Duration Caused Gradually Severer IDD

We also hypothesized that compression duration was another critical factor to determine the severity of IDD. With radiological analysis, we observed that the narrower intervertebral height was found with increased compression duration, as depicted in Figure 4(a). In histological result of Figure 4(b), IVDs showed a gradual severity of degeneration after 3-, 7-, and 14-day constant compression under the mild compression pressure. For sham surgery group, the IVD showed as normal morphology of nucleus pulposus (NP) and organized annulus fibrosus (AF) with discrete fibrous lamellae. By contrast, compression with 3 days induced shrunken NP with slight proliferated chondrocytes and small fibrosus tissue and with slight disorganized AF. When IVD was compressed for 7 days, the area of NP significantly decreased with remarkable proliferated chondrocytes and lager fiber bundles, and morphology of AF obvious changed with disorganized, tear lamellar. Finally, at 14 days of compression, this resulted in disappearance of NP and AF, which was replaced by fibrosus tissue and the dislocation of the two vertebrae.

The article "Intervertebral Disc Degeneration and Low Back Pain Depends on Duration and Magnitude of Axial Compression" was published in 2022. Journal: Oxid Med Cell Longev.

Similar to compression magnitude, gradient compression duration also led to a decrease of ECM of collagen II and aggrecan, and an increase of catabolic factors of IL-1*β* and MMP3, as depicted in Figure 4(c) with western blot analysis. In addition, IHC examination suggested the expression of collagen II and aggrecan gradually decreased in accordance with the increase of compression time, as depicted in Figure 4(d). Therefore, compression duration was another factor to affect IDD.

## 4. Discussion

In this study, when NPCs suffered gradual increased mechanical stress, the cells exhibited gradual downregulated expression of ECM-related gene of aggrecan, upregulated expression of IDD-related gene of MMP3, and LBP-related gene of CGRP and SP, suggesting a significant IDD and LBP in vitro. Additionally, mechanical stress-induced IVDs had gradient degeneration in accordance with the increase of stress duration or magnitude, showing as decrease of intervertebral heights, destruction of IVD anatomy, decrease of ECM, and increase of catabolic factors. Therefore, we made reasonable conclusion that axial mechanical stress was the key pathological factor to initiate IDD and related LBP in a dose-response manner.

We reported a measurable Ilizarov-type axial compression apparatus for coccygeal single IVD in mice. Previous studies also reported some compression devices in rodent, but there were disadvantages for them. There had previously been no method to directly quantify the compression force. This resulted in difficulty in quantification of fixed comparison gradation among different groups [13]. In addition, targeting single levels of IVD provided more stable and comparable results than that for multiple levels [14]. Finally, the pressure in the four directions perpendicular to each other can ensure that the IVD is evenly stressed; otherwise, there would be shear stress when the intervertebral disc is pressurized without four directions [15].

The article "Intervertebral Disc Degeneration and Low Back Pain Depends on Duration and Magnitude of Axial Compression" was published in 2022. Journal: Oxid Med Cell Longev.

The pathophysiological mechanism of axial stress for IDD may be combined. First, continuous excessive axial compress may cause direct physical damage for IVD, suggesting as the squeeze of NP and tear of AF. Second, the excessive compress may further cause the change of biochemical environment in IVD. For example, nucleus pulposus cells (NPCs) would secrete plenty of inflammatory or catabolic factors to catalyze the cascade of damage of IVD [16]. Also, the function of NPCs to maintain homeostasis, for example, the secretion of collagen II and aggrecan, would be interfered when they suffer excessive axial loading [16]. Finally, the programmed cell death caused by excessive loading may be another reason for IDD [17].

Although rodents are suitable to act as mechanical models of the human lumbar disc [18], the mouse-related IDD models were rare, especially that some studies related to gene function have to be verified in gene-knockout mouse. The traditional puncture-induced IDD, however, is difficult for operation in mouse IVD due to the diameter of the mouse's tail, which is only 2–3 mm. Some authors also proposed the tail-bending model to induce IDD; however, the model is difficult to quantify for comparison, and the IVD cannot bear much pressure [19]. The model we report here is easy to quantify the pressure and effective to induce IDD with different severity levels (e.g., mild, moderate, and severe) and provides a convenient method for IVD-related research in gene-knocked mice.

## 5. Conclusions

In conclusion, IDD and LBP had strong correlation with axial compression and the severity depended on duration and magnitude of compression, showing as a dose-response manner. In addition, the Ilizarov-type compression apparatus was useful for study about IVDs in mice, which provides a convenient method for further IVD-related research of mice.

## Figures and Tables

**Figure 1:** Mechanical stress caused gradual IDD and LBP in NPCs. (a, b) NPCs exhibited gradual downregulated expression of ECM-related gene of aggrecan and upregulated expression of IDD-related gene of MMP3, with a time-response manner. (c, d) NPCs had significantly upregulation of LBP-related gene of CGRP and substance P, with a time-response manner. (The data are shown as mean ± SD. ∗<0.05, ∗∗<0.01, and ∗∗∗<0.001when compared among each group. One-way ANOVA and Tukey's HSD multiple comparison test were used for statistical analysis).

**Figure 2:** Illustration of Ilizarov-type compression apparatus in IVD of mouse. (a). Schematic image of an Ilizarov-type coccygeal IVD compression apparatus. (b). General images of an Ilizarov-type compression apparatus produced 400 g axial stress for Co7-8 in the tail of mouse. The force between each springs and the ring was fixed at the same level in turn with sensors. (c). Lateral X-ray evaluation after installation of apparatus.

The article "Intervertebral Disc Degeneration and Low Back Pain Depends on Duration and Magnitude of Axial Compression" was published in 2022. Journal: Oxid Med Cell Longev.

**Figure 3:** Radiological and histological evaluation of IDD with gradient compression magnitude. (a) X-ray examination showed a gradual narrowing of the intervertebral height in accordance with the severity level of compression pressure. Arrows indicated the targeted IVDs. (b) H-E staining also suggested a gradual severer IDD along with severer compression pressure. (c) Western blot analysis suggested a gradient compression magnitude induced by a gradual decrease of collagen II and aggrecan and increase of IL-1*β* and MMP3. (d) IHC staining indicated the distribution and content of collagen II and aggrecan decreased along with gradient compression magnitude (the data are shown as mean ± SD. *N* = 3-5 for each group. ∗<0.05, ∗∗<0.01, and ∗∗∗<0.001 when compared among each group. One-way ANOVA and Tukey's HSD multiple comparison test were used for statistical analysis).

**Figure 4:** Radiological and histological analysis in IDD with gradient compression duration. (a) A gradually narrower intervertebral height in accordance with longer compression duration. White arrows indicated the targeted IVDs. (b) A gradually more severe IDD, along with severer compression pressure, as shown in H-E staining. (c) Western blot analysis suggested that gradient compression magnitude induced a gradual decrease of collagen II and aggrecan and an increase of IL-1*β* and MMP3. (d) IHC staining indicated the distribution and content of collagen II and aggrecan remarkable decrease with gradient compression magnitude (the data are shown as mean ± SD. *N* = 3-5 for each group. ∗<0.05, ∗∗<0.01, and ∗∗∗<0.001 when compared among each group. One-way ANOVA and Tukey's HSD multiple comparison test were used for statistical analysis).

## Data Availability

The data that support the findings of this study are available from the corresponding author upon reasonable request.

## Abbreviations

IDD: Intervertebral disc degeneration
LBP: Low back pain
IVD: Intervertebral disc
NP: Nucleus pulposus
AF: Annulus fibrosus
NPCs: Nucleus pulposus cells.

## References

[1] Modic M. T., Ross J. S. (2007). Lumbar degenerative disk disease. *Radiology*.

[2] Vergroesen P. P., Kingma I., Emanuel K. S. (2015). Mechanics and biology in intervertebral disc degeneration: a vicious circle. *Osteoarthritis and Cartilage*.

[3] Kawaguchi Y. (2018). Genetic background of degenerative disc disease in the lumbar spine. *Spine Surg Relat Res*.

[4] Jiao Y., Lin Y., Zheng Y., Yuan Y., Chen Z., Cao P. (2019). The bacteria-positive proportion in the disc tissue samples from surgery: a systematic review and meta-analysis. *European Spine Journal*.

The article "Intervertebral Disc Degeneration and Low Back Pain Depends on Duration and Magnitude of Axial Compression" was published in 2022. Journal: Oxid Med Cell Longev.

[5] Battié M. C., Videman T., Gibbons L. E., Fisher L. D., Manninen H., Gill K. (1995). 1995 Volvo Award in clinical sciences. Determinants of lumbar disc degeneration. A study relating lifetime exposures and magnetic resonance imaging findings in identical twins. *Spine*.

[6] Muraki S., Oka H., Akune T. (2009). Prevalence of radiographic lumbar spondylosis and its association with low back pain in elderly subjects of population-based cohorts: the ROAD study. *Annals of the Rheumatic Diseases*.

[7] Malik K. M., Cohen S. P., Walega D. R., Benzon H. T. (2013). Diagnostic criteria and treatment of discogenic pain: a systematic review of recent clinical literature. *The Spine Journal*.

[8] Chou R., Qaseem A., Snow V. (2007). Diagnosis and treatment of low back pain: a joint clinical practice guideline from the American College of Physicians and the American Pain Society. *Annals of Internal Medicine*.

[9] Chen Z., Jiao Y., Zhang Y., Wang Q., Wu W. (2022). *G-protein coupled receptor 35 induces intervertebral disc degeneration by mediating the influx of calcium ions and upregulating reactive oxygen species*. *Oxidative Medicine and Cellular Longevity*.

[10] Lotz J. C., Chin J. R. (2000). Intervertebral disc cell death is dependent on the magnitude and duration of spinal loading. *Spine*.

[11] Zheng J., Zhang J., Zhang X., Guo Z., Wu W. (2021). Reactive oxygen species mediate low back pain by upregulating substance P in intervertebral disc degeneration. *Oxidative Medicine and Cellular Longevity*.

[12] Choi H., Tessier S., Silagi E. S. (2018). A novel mouse model of intervertebral disc degeneration shows altered cell fate and matrix homeostasis. *Matrix Biology*.

[13] Yan Z., Pan Y., Wang S. (2017). Static compression induces ECM remodeling and integrin *α*2*β*1 expression and signaling in a rat tail caudal intervertebral disc degeneration model. *Spine*.

[14] Papuga M. O., Proulx S. T., Kwok E. (2010). Chronic axial compression of the mouse tail segment induces MRI bone marrow edema changes that correlate with increased marrow vasculature and cellularity. *Journal of Orthopaedic Research*.

[15] Guo J. B., Che Y. J., Hou J. J. (2020). Stable mechanical environments created by a low-tension traction device is beneficial for the regeneration and repair of degenerated intervertebral discs. *The Spine Journal*.

[16] Sowa G. A., Coelho J. P., Bell K. M. (2011). Alterations in gene expression in response to compression of nucleus pulposus cells. *The Spine Journal*.

[17] Huang D., Peng Y., Ma K. (2020). Puerarin relieved compression-induced apoptosis and mitochondrial dysfunction in human nucleus pulposus mesenchymal stem cells via the PI3K/Akt pathway. *Stem Cells International*.

The article "Intervertebral Disc Degeneration and Low Back Pain Depends on Duration and Magnitude of Axial Compression" was published in 2022. Journal: Oxid Med Cell Longev.

[18] Elliott D. M., Sarver J. J. (2004). Young investigator award winner: validation of the mouse and rat disc as mechanical models of the human lumbar disc. *Spine*.

[19] Court C., Chin J. R., Liebenberg E., Colliou O. K., Lotz J. C. (2007). Biological and mechanical consequences of transient intervertebral disc bending. *European Spine Journal*.

